# High Blood Pressure Prevalence and Significant Correlates: A Quantitative Analysis from Coastal Karnataka, India

**DOI:** 10.5402/2013/574973

**Published:** 2012-12-03

**Authors:** Chythra R. Rao, Veena G. Kamath, Avinash Shetty, Asha Kamath

**Affiliations:** Department of Community Medicine, Kasturba Medical College, Manipal University, Manipal 576104, Karnataka, India

## Abstract

Hypertension is a premier risk factor for cardiovascular disease which can be recognized if sought and treated effectively. Effective management of high blood pressure is possible when the magnitude of the problem is identified. So, a cross-sectional community based survey among 1,239 respondents aged ≥30 years was designed to estimate the prevalence and the sociodemographic correlates of hypertension among adults aged ≥30 years. Data was collected by personal interviews, followed by anthropometric and blood pressure measurements. Analysis was done using Statistical Package for the Social Sciences (SPSS) version 11.5. The prevalence of hypertension was 43.3%, with the prevalence being more among males (51.6%) as compared to females (38.9%). Of the total prevalence 23.1% (287) were known cases, and 20.2% (250) were newly detected cases. Based on the seventh report of the Joint National Committee (JNC VII) on high blood pressure, prehypertension was noted among 38.7%. Advancing age, male gender, current diabetic status, central obesity, overweight and obesity as defined by body mass index, and family history of hypertension were identified as significant correlates for hypertension by multivariate logistic regression.

## 1. Introduction

Hypertension (HTN) is an enormous health problem and is one of the biggest health challenges in the 21st century. Although the condition is common, readily detectable, and easily treatable, it is usually asymptomatic and often leads to lethal complications if left untreated [1]. The Global Burden of Disease study has reported HTN as the 4th contributor to premature death in developed countries and the 7th in the developing countries [2]. Analysis of worldwide data on global burden of HTN showed an overall prevalence of 26.4% among the adult population in 2000 [3]. In India, the prevalence of HTN ranges between 20%–40% in urban areas and 12%–17% among rural adults [4]. 

India, being a culturally and socially diverse nation, differences would be noted in the region-wise prevalence of hypertension, but research regarding the same is inadequate in coastal Karnataka. This inadequacy necessitated us to conduct this study with the objective of assessing the prevalence of hypertension and study the sociodemographic correlates of hypertension. 

## 2. Methods

A cross-sectional community-based survey was conducted among individuals of either sex, aged 30 years and above. The study was carried out in the field practice area of the Department of Community Medicine, Kasturba Medical College, Manipal in coastal Karnataka, a Southern state of India. The field practice area covers a population of 45,587 individuals living in 7,164 families spread out in 11 villages. The population in these villages is homogeneous in terms of occupation, socioeconomic status, and food habits.

### 2.1. Sample

Institutional ethical clearance was obtained prior to initiation of the study. Study population included all men and women aged 30 years and above. Pregnant or lactating women up to 12 weeks after partum were excluded from the study, due to possible variations in blood pressure during this period.

Considering a prevalence of 14% for rural adults, with an allowable error of 15% and 95% confidence level, the sample size estimated was 1,092. A nonresponse rate of 20% required a sample of 1,310 to be studied. The detailed methodology of selection of subjects has been described earlier [5]. Written informed consent was obtained from all the subjects.

### 2.2. Sociodemographic Variables and Risk Factors

During house visits, the objectives of the study were explained to the eligible household members, and data was collected by personal interviews using a predesigned questionnaire. The questionnaire included details on sociodemographic variables, past/family history of hypertension, and physical activity status [6]. Socioeconomic status was assessed using modified Uday-Parikh scale. Following this, anthropometric measurements and blood pressure were recorded.

Weight was recorded using a standard weighing scale (Krups weighing scale, New Delhi, India) kept on a firm horizontal surface. Weight was recorded to the nearest 500 gm. Height was recorded using a measuring tape to the nearest 1 cm. Subjects were requested to stand upright, without shoes, with their back against the wall, heels together and looking forward. Body mass index (BMI) was calculated using the formula of weight (kg)/height (m^2^). Waist circumference was measured to the nearest 0.1 cm at the midpoint between costal margin and iliac crest using a nonstretchable measuring tape. Hip circumference was measured at the level of the greater trochanters (widest portion of the hip) to the nearest 0.1 cm by a measuring tape. Waist-hip ratio was calculated as the ratio of waist circumference over hip circumference [7]. 

A person was considered to be obese if body mass index ≥30 kg/m^2^ and overweight when BMI ≥ 25 kg/m^2^. Central/abdominal obesity was considered to be present when waist circumference ≥94 cm in males and ≥80 cm in females. Waist-hip ratio >1 for males and >0.85 for females was defined as truncal obesity [8, 9].

Blood pressure was measured in right arm in sitting posture, with the subject in a relaxed state. Standardized mercury sphygmomanometer (Diamond Deluxe BP Apparatus, Pune, India) with adult size cuff was used. The first appearance of (phase 1 of Korotkoff sounds) sound was used to define systolic blood pressure (SBP). The disappearance of sound (phase 5) was used to define diastolic blood pressure (DBP). Two readings were taken five minutes apart, and the average of the two readings was taken as the final blood pressure reading. A person was considered to be a hypertensive if he/she was an already diagnosed case of hypertension and/or on treatment or had current SBP ≥ 140 mm of Hg and/or DBP ≥ 90 mm of Hg (the seventh report of the Joint National Committee on prevention, detection, evaluation, and treatment of high blood pressure, JNC VII criteria) [10].

Blood sugar estimation was done for all the subjects using a glucometer. A person was considered to be a diabetic if he/she was an already diagnosed case of diabetes and/or on treatment or had current fasting capillary blood glucose ≥110 mg/dL (fasting being defined as no caloric intake for at least 8 hours) [11]. 

Individuals with either a parent or a sibling (brother or sister) having hypertension were considered to have a positive family history. Eligible subjects unavailable during the first house visit were approached on another preinformed date as per their convenience. Even after two such visits if the subject was noncompliant, then he/she was considered as a nonrespondent.

### 2.3. Statistical Analysis

All statistical analyses were performed using Statistical Package for Social Sciences (SPSS) version 11.5. Prevalence and risk factors of hypertension are presented as percentages. The association between hypertension and sociodemographic variables, diabetes, obesity, physical activity, and family history of hypertension was assessed by comparing the prevalence of hypertension in individuals with and without these risk factors. The chi-square test was used to analyze the differences, considering a *P* < .05 as statistically significant. The odds ratios (ORs) of the statistically significant variables detected in the univariate analysis and their 95% confidence intervals were calculated. A multiple logistic regression analysis was carried out to obtain adjusted odds ratios for the variables. All the variables having a *P* < .2 in the univariate analysis were included in the multiple logistic regression analysis, with hypertension as a dichotomous outcome and age, sex, socioeconomic status, physical activity, positive family history of hypertension, current diabetic status, BMI, and central obesity as independent variables. Variables with significant adjusted odds ratios (*P* < .05) were considered to be independently associated with hypertension.

## 3. Results

### 3.1. Baseline Characteristics of the Sample

The baseline characteristics of the study subjects are shown in Table 1. The study included 1,419 subjects with a response rate of 87.3%. The total sample studied was 1,239, of which 434 (35%) were males and 805 (65%) were females. Males in the study area were not available during the survey as they were either employed overseas or in the neighbouring states or were involved in occupations such as fishing and unskilled daily wage labour. Of the total study subjects, 85.6% were Hindus, 8.6% Muslims, and 5.7% Christians. The literate proportion in the sample was 81.2%. Socioeconomic status for rural areas assessed by modified Uday-Parikh scale showed that 70.1% belonged to middle class, 27.6% to lower class, and 2.3% to upper class. Sedentary life style was observed in 11.1% of the subjects, while 41.8% were engaged in moderate physical activity. Family history of hypertension was present among 41% of the individuals. In the study, 21.4% of the subjects were overweight, while 6.6% of the individuals were found to be obese when BMI was used as the defining criteria, but over half of the subjects had abdominal and truncal obesity (51.7% and 62.1% resp.). Among the study subjects, 16% had diabetes. This included the proportion of individuals already diagnosed with diabetes and/or on treatment along with previously normal individuals who had fasting capillary blood glucose ≥110 mg/dL, tested using a glucometer at the time of the conduct of the study.

### 3.2. Prevalence of Hypertension

The prevalence of hypertension was 43.3% of which 20.2% were previously undiagnosed cases. A higher prevalence was noted among males (51.6%) as compared to females (38.9%), as shown in Table 2, which was statistically significant (chi-square = 18.61, *P* value  <  .001).

### 3.3. Association between Hypertension and Study Variables

The blood pressure recording of the study subjects classified according to JNC VII criteria with respect to age has been described in Table 3. The number of individuals in the normotension and prehypertension category were more in the younger age groups, while the prevalence of stage 1 and stage 2 hypertension was higher in the older subjects. Prehypertensives constituted 38.7% of the study subjects, highlighting the need for screening of individuals beginning at age of 30 years or earlier. Statistical significance was noted between hypertension and advancing age of the subjects (*χ*_trend_^2^ = 113.93, *P* < .001, df = 1).

Advancing age, male gender, current diabetic status, overweight and obesity defined by BMI, and central obesity identified in the univariate analysis were also found to have significant association with hypertension in multivariate analysis, as shown in Table 4.

## 4. Discussion

The World Health Report 2002 identified high blood pressure (BP) as one of the five important risk factors for noncommunicable diseases worldwide. It is estimated that elevated BP alone causes about 50% of cardiovascular disease (CVD) worldwide. It is important to emphasize that while 10–30% of adults worldwide suffer from high BP as currently defined by the JNC VII report, an additional 50%–60% could improve their prognosis if they had lower BP [12]. A downward shift of about two mm Hg in the blood pressure distribution of the general population should result in an annual reduction by about 6% in stroke, 4% in coronary heart disease, and 3% in all-cause mortality. Similarly, studies have reported that a 2-3 mm Hg average reduction in individuals with high normal blood pressure should result in a 20%–25% decrease in the incidence of hypertension. Therefore, great emphasis must be placed on primary prevention of hypertension in the population [13].

The prevalence of hypertension was found to be high in the present study (43.3%), as compared to other reported literature, but was comparable to that of Kerala, which is similar to our coastal study area with respect to diet, occupation, and high literacy levels [14, 15]. Cross-sectional data on hypertension prevalence vary with respect to selection of study subjects, sample size, and defining criteria. Most of the studies report a prevalence ranging between 20%–30% [16–22]. The higher prevalence noted among males and the agewise distribution noted in the study were concordant with other reported literature [14, 20, 23, 24]. Advancing age, male gender, current diabetic status, overweight and obesity defined by BMI, and central obesity were identified as significant correlates in the study, based on multivariate analysis, which was in conformity with studies done in India and abroad [19, 20, 23, 25–28].

A community-based study has the inherent limitation of resource constraints in terms of manpower, which is acceptable to the population. So, blood pressure measurements were taken during a single visit and repeated measurements on different occasions and different settings could not be done. But, estimation of blood pressure was done by a single trained investigator in order to have a uniform pattern of blood pressure measurement. The authors do agree that there was a poor representation of males, and an attempt to quantify life style changes was not made in the present study. Although we accept these shortcomings, it is also true that this study was planned to quantify the problem of hypertension in the community, so that future interventions could be planned based on the existing level of the risk factor in the study population. There were no earlier data on prevalence of hypertension, in the area, which necessitated us to conduct this study. The methodology was fairly rigorous and the sample size was also sufficiently large. The high prevalence of hypertension, noted in the study, necessitates the need to plan future community-based studies in the same region with an additional objective to quantify the lifestyle factors responsible for the same. Stress, staying away from home due to being overboard on the boats for fishing purposes, odd hours of work with changed sleep pattern, consumption of salted fish, less physical activity predisposing to obesity, and probable indulgence in usage of tobacco and alcohol to beat loneliness could be some of the potential reasons for the high prevalence of hypertension noted in the area, as speculated by the authors. Central obesity was found to be present in a substantial proportion of the population, which points towards the need for lifestyle modifications in order to reduce this risk factor. Research into the underlying mechanisms may have policy implications to address the problem of hypertension.

## 5. Conclusion

A significant number of individuals were identified to be in the prehypertension category, stressing the need to initiate screening strategies at an earlier age and promote opportunistic screening for hypertension during routine health care visits, so that major health gains can be made through the implementation of primary prevention strategies.

## Figures and Tables

**Table 1:** Characteristics of the study subjects.

Variables	Males	Females	Total
	no. (%)	no. (%)	no. (%)
	*n* = 434	*n* = 805	*n* = 1239
Age group (yrs.)			
30–39	115 (26.5)	252 (31.3)	367 (29.6)
40–49	123 (28.4)	183 (22.8)	306 (24.6)
50–59	77 (17.7)	138 (17.1)	215 (17.4)
≥60	119 (27.4)	232 (28.8)	351 (28.4)
Occupation*			
Heavy	82 (18.9)	219 (27.3)	301 (24.4)
Moderate	235 (54.1)	580 (72.0)	815 (65.7)
Sedentary	117 (27.0)	6 (0.7)	123 (9.9)
BMI**			
<24.9	316 (72.8)	576 (71.6)	892 (72.0)
25.0–29.9	92 (21.2)	173 (21.5)	265 (21.4)
≥30.0	26 (6.0)	56 (6.9)	82 (6.6)
Waist and hip measurements			
Central obesity	78 (18.0)	562 (69.8)	640 (51.7)
Truncal obesity	58 (13.4)	711 (88.3)	769 (62.1)
Presence of Diabetes	82 (18.8)	116 (14.4)	198 (16.0)

*Occupation—heavy: unskilled; moderate: housewives, skilled, and service jobs; Sedentary: unemployed/retired.

**Body Mass Index (kg/m^2^).

**Table 2:** Gender-wise prevalence of hypertension in the study population.

Hypertension	Males	Females	Total
	no. (%)	no. (%)	no. (%)
	*n* = 434	*n* = 805	*n* = 1239
Known cases	97 (22.4)	190 (23.6)	287 (23.2)
Newly detected cases	127 (29.3)	123 (15.3)	250 (20.2)

Total hypertension	224 (51.6)	313 (38.9)	537 (43.3)

**Table:** (a) Classification of blood pressure according to JNC VII* criteria

Blood pressure	30–39 yrs.	40–49 yrs.	50–59 yrs.	≥60 yrs.	Total
	no. (%)	no. (%)	no. (%)	no. (%)	no. (%)
	*n* = 367	*n* = 306	*n* = 215	*n* = 351	*n* = 1239
Normotension	145 (39.5)	93 (30.4)	40 (18.6)	51 (14.5)	329 (26.6)
Prehypertension	157 (42.8)	117 (38.2)	86 (40.0)	119 (33.9)	479 (38.7)
Stage 1 hypertension	45 (12.3)	64 (20.9)	55 (25.6)	106 (30.2)	270 (21.8)
Stage 2 hypertension	20 (5.4)	32 (10.5)	34 (15.8)	75 (21.4)	161 (13.0)

Chi-square for trend (*χ*_trend_^2^) = 113.93, *P* < .001, df = 1.

*JNC VII classification of blood pressure.

**Table:** (b) *JNC VII classification of blood pressure

Category	Systolic blood pressure (SBP) mm Hg		Diastolic blood pressure (DBP) mm Hg
Normal	<120	and	<80
Prehypertension	120–139	or	80–89
Hypertension Stage 1	140–159	or	90–99
Hypertension Stage 2	≥160	or	≥100

**Table 4:** Summary table of significant correlates for hypertension.

Variable	*n*	%	(95% CI)	Crude OR	(95% CI)	Adjusted OR	(95% CI)
Age group (yrs.)*							
30–39	367	18.3	(14.3–22.3)	1.00	(1.00)	1.00	(1.00)
40–49	306	36.6	(31.2–42.0)	**2.58**	**(1.81–3.67)**	**2.33**	**(1.59–3.42)**
50–59	215	53.0	(46.3–59.7)	**5.05**	**(3.46–7.36)**	**4.73**	**(3.10–7.24)**
≥60	351	69.5	(64.7–74.3)	**10.21**	**(7.20–14.47)**	**9.90**	**(6.47–15.13)**

Gender*							
Male	434	51.6	(46.9–56.3)	**1.67**	**(1.32–2.12)**	**2.84**	**(1.97–4.09)**
Female	805	38.9	(35.5–42.3)	1.00	(1.00)	1.00	(1.00)

Literacy*							
Illiterate	233	58.8	(52.5–65.1)	1.00	(1.00)	1.00	(1.00)
Primary (1st–4th class)	196	48.0	(41.0–55.0)	0.64	(0.44–0.94)	0.63	(0.39–1.01)
Secondary (5th–12th class)	734	37.6	(34.1–41.1)	0.42	(0.31–0.57)	0.55	(0.35–0.76)
Graduation and above	76	39.5	(28.5–50.5)	0.45	(0.26–0.77)	0.67	(0.34–1.31)

Currently diabetic*							
Yes	198	68.2	(61.7–74.7)	**3.40**	**(2.46–4.71)**	**1.52**	**(1.04–2.23)**
No	1041	38.6	(35.6–41.6)	1.00	(1.00)	1.00	(1.00)

Body Mass Index (kg/m^2^)*							
<24.9	892	37.8	(34.6–41.0)	1.00	1.00	1.00	1.00
25.0–29.9	265	55.1	(49.1–61.1)	**2.02**	**(1.53–2.66)**	**2.05**	**(1.50–3.09)**
≥30	82	65.9	(55.6–76.2)	**3.17**	**(1.97–5.11)**	**3.22**	**(1.80–5.77)**

Central obesity*							
Yes	640	48.8	(44.9–52.7)	1.58	(1.26–1.98)	1.77	(1.21–2.59)
No	599	37.6	(33.7–41.5)	1.00	(1.00)	1.00	(1.00)

Socioeconomic status							
Low	342	44.7	(39.4–50.0)	1.00	(1,00)	—	—
Middle	869	42.5	(39.2–45.8)	0.91	(0.70–1.17)	—	—
High	28	53.6	(35.1–72.1)	1.42	(0.65–3.08)	—	—

Family history of hypertension							
Yes	512	45.1	(40.8–49.4)	0.97	(0.76–1.24)	**1.42**	**(1.05–1.92)**
No	727	42.1	(38.5–45.7)	1.00	(1.00)	1.00	(1.00)

Physical activity*							
No	137	71.5	(63.9–79.1)	3.79	(2.56–5.60)	—	—
Yes	1102	39.8	(36.9–42.7)	1.00	(1.00)	—	—

*P < .001 by chi-square test.
